# Expression and the Prognostic Value of Biglycan in Gastric Cancer

**DOI:** 10.1155/2022/2656480

**Published:** 2022-09-06

**Authors:** Sizhe Hu, Peipei Li, Chenying Wang, Xiyong Liu

**Affiliations:** ^1^Department of Gastrointestinal Surgery, Affiliated Dongyang People's Hospital of Wenzhou Medical University, Dongyang, Zhejiang 322100, China; ^2^School of Medicine, Zhejiang University City College, Hangzhou, Zhejiang 310015, China; ^3^Sino-American Cancer Foundation, Covina, CA 91722, USA

## Abstract

**Background:**

Biglycan (BGN) is a family member of small leucine-rich repeat proteoglycans. High expression of BGN might enhance the invasion and metastasis in some types of tumors. Here, the prognostic significance of BGN was evaluated in gastric cancer. *Material and Methods*. Two independent Gene Expression Omnibus (GEO) gastric cancer microarray datasets (*n* = 64 and *n* = 432) were collected for this study. Kaplan-Meier analysis was applied to evaluate if BGN impacts the outcomes of gastric cancer. Protein-protein interaction (PPI) analysis was performed on gastric cancer-related genes and BGN targets, and those interactions with confidence interval (CI) ≥ 0.7 were chosen to construct a PPI network. The gene set enrichment analysis (GSEA) was used to explore BGN and cancer-related gene signatures. Gene Transcription Regulation Database (GTRD) and ALGGEN-PROMO predicted the transcription factor binding sites (TFBSs) of the BGN promoter. BGN protein level in gastric cancer tissue was determined by immunohistochemistry (IHC). Bioinformatic analysis predicted the putative TFs of BGN.

**Results:**

For gastric cancer, the mRNA expression level of BGN in tumor tissue was significantly higher than that in normal tissue. Kaplan-Meier analysis showed that higher expression of BGN mRNA was significantly associated with more reduced recurrence-free survival (RFS). GSEA results suggested that BGN was significantly enriched in gene signatures related to metastasis and poor prognosis, revealing that BGN might be associated with cell proliferation, poor differentiation, and high invasiveness of gastric cancer. Meanwhile, the putative TFs, including AR, E2F1, and TCF4, were predicted by bioinformatic analysis and also significantly correlated with expression of BGN in mRNA levels.

**Conclusion:**

High expression of BGN mRNA was significantly related to poor prognosis, which suggested that BGN was a potential prognostic biomarker and therapeutic target of gastric cancer.

## 1. Introduction

Gastric cancer is the sixth most common malignant tumor and is the second leading cause of cancer-induced death in the world [1]. In East Asia (China, Japan, and Korea), the incidence of gastric cancer is higher than in other areas over the world [2]. It was estimated that about one million new cases of gastric cancer were diagnosed globally in 2018, and about half of the new cases occurred in China [3]. The 5-year overall survival of gastric cancer is only 20% to 30% due to cancer progression [4], although numerous new treatments have been utilized, including but not limited to chemotherapy, targeted therapy, and immunotherapy. However, for early gastric cancer, the 5-year overall survival is more than 90% [5]. Unfortunately, early-stage gastric cancer usually has no or only nonspecific symptoms. Thus, the appearance of symptoms usually suggests the advanced gastric cancer. Gastroscopy is a routine screening method for gastric cancer, but it is not widely accepted because it is invasive [6]. Currently, several tumor markers are used in the clinic for early detection of gastric cancer. These markers include carcinoembryonic antigen (CEA), pepsinogen, *α*-fetoprotein (AFP), carbohydrate antigens (CA), CA72-4, CA125, and CA24-2. However, the sensitivity and specificity of these serum indicators are poor [7]. Thus, it is urgently needed to explore novel biomarkers for early diagnosis and prognosis prediction for gastric cancer patients.

Biglycan (BGN) is a family member of small leucine-rich repeat proteoglycans (SLRPs) characterized by a core protein with leucine-rich repeats [8]. Initially, BGN was only considered as a component maintaining the structural integrity of the extracellular matrix (ECM) and involved in the regulation of inflammatory response, skeletal muscle development, and regeneration [9, 10]. In a decade, it was found that BGN is a signal molecule, playing an essential role in angiogenesis, cell proliferation, differentiation, and migration [11–13]. In recent years, it has been gradually found that BGN is highly expressed in various malignant tumors, such as endometrial cancer [14], ovary cancer [15], pancreatic adenocarcinoma [16], esophageal squamous cell carcinoma [17], colorectal cancer [18], and gastric cancer [19], suggesting an essential role of BGN in the pathogenesis and progression of cancer. In some types of these cancers, high expression of BGN enhances the ability of invasion and metastasis of tumor cells [18–20] or contributes to poor prognosis [16, 17, 21, 22].

Therefore, BGN is closely related to the occurrence and development of a variety of tumors and is a potential target molecule for tumor treatment. The purpose of the present study is to verify the BGN expression and the prognostic value of BGN in gastric cancer. In this study, we investigated the prognostic value of BGN in gastric cancer by involving an external transcriptome data set from the TCGA database. To understand the role of BGN in gastric cancer, we analyzed our tissue microarray, including 125 cases of gastric cancers, for immunohistochemical BGN expression.

## 2. Materials and Methods

### 2.1. Microarray Gene Expression Datasets

Two independent Gene Expression Omnibus (GEO) gastric cancer microarray datasets (total *n* = 496) were collected for this study. There were 432 cases of gastric cancer patients from South Korea in GSE26253 dataset [23], and all participants had clinical and follow-up annotations. GSE65801 [24] contained 32 Chinese patients but had no follow-up annotations. Detailed information about the two downloaded datasets is listed in Table 1. To normalize the mRNA expression levels in the GSE26253 dataset, we restratified BGN scores into four grades (Q1, Q2, Q3, and Q4) based on the percentile. Low-BGN score grades (Q1+Q2) and high-BGN score grades (Q3+Q4) were also divided by the median value of gene expression.

The recurrence-free survival (RFS) period was defined as the time from initial surgery until tumor recurrence. Kaplan-Meier survival plot was used to display the proportion of the population's RFS by the length of follow-up.

### 2.2. Gene Set Enrichment Analysis (GSEA)

The GSEA software v3.0 was downloaded from http://www.broad.mit.edu/gsea and run on the Java 8.0 platform [25]. All dataset (.gct) and phenotype label (.cls) files were created and loaded into the GSEA software, and gene sets were updated from the above website. The detailed protocol could see in our previous publications [26]. Here, the permutation number was 1,000, and the phenotype label was ILMN_2206746 (BGN).

### 2.3. Data Management and Statistical Methods

Student's *t*-test, one-way analysis of variance (ANOVA), and nonparametric tests were used to test differences among subgroups for continuous data. The Pearson Chi-square and likelihood test was used for categorical data analyses. Kaplan-Meier analysis was used to estimate the proportion of the population's RFS by the length of follow-up in months. Hazard ratios (HRs) [21] with 95% confidence intervals (CI) were calculated using Cox proportional hazard regression analysis. Two-sided *p* values less than 0.05 were considered statistically significant. The R and JMP statistical software were used for the above analysis unless otherwise noted.

### 2.4. Eligible Transcription Factor (TF) Prediction

The promoter region of the BGN gene was visualized on http://genome.ucsc.edu/cgi-bin/hgGateway. The signal of H3K4Me3 was used to localize the promoter region. The TF binding sites (TFBSs) of BGN promoter were predicted by Gene Transcription Regulation Database (GTRD) (http://gtrd.biouml.org/) and ALGGEN-PROMO (http://alggen.lsi.upc.es/cgi-bin/promo_v3/promo/promoinit.cgi?dirDB=TF_8.3).

### 2.5. Immunohistochemistry (IHC) Assays of Tissue Microarray

The protocol for the use of human tissue was approved by the Institutional Review Board [13] of the Affiliated Dongyang People's Hospital of Wenzhou Medical University (Zhejiang, China). Before the study, all patients gave their written informed consent to allow us to use left tissue samples for scientific research. All eligible participants had received radical gastrectomy or palliative gastrectomy. The primary tumor samples were obtained from surgical specimens. The exclusion criteria of participants were those with (1) no informed consent signed and (2) multiple cancers. A total of 125 pairs of gastric cancer specimens, including cancerous tissue and adjacent normal tissue, that underwent surgery in 2018, were eventually enrolled. The above-mentioned tissue specimens were fixed in ethanol at 4°C for 1 h, followed by paraffin embedding. Thereafter, specimens were sliced with a microtome into 4 *μ*m sections. These sections were cultivated with 3% H_2_O_2_ at room temperature for 5-10 min to eradicate the activity of endogenous peroxidase, followed by 10 min of block with bovine serum albumin (BSA). The primary antibody working solution was then added dropwise followed by a 1-2 h cultivation at 37°C or an overnight one at 4°C. Phosphate-buffered saline (PBS) was introduced to rinse sections 3 times. Subsequently, the secondary antibody working solution was also introduced dropwise, and the system was incubated at 37°C for 10-30 min. Antibodies involved were as follows: anti-rabbit BGN (1 : 2000, ab209234, Abcam, UK) and goat anti-rabbit IgG (1 : 500, ab150077, Abcam, UK). The previously described protocols of deparaffinization and immunohistochemistry (IHC) staining were used to apply to the multiple-tissue array [27].

## 3. Results

### 3.1. The Prognostic Significance of BGN for Gastric Cancer

In the GSE65801 dataset, we came to the same conclusion that BGN mRNA level was higher in tumor tissue than the normal tissue (Figure 1(a)). Kaplan-Meier analysis showed that higher expression of BGN was significantly associated with poorer RFS in gastric cancer patients. In the GSE26253 dataset, samples were divided into four subgroups, Q1, Q2, Q3, and Q4, according to the expression level of BGN. BGN mRNA levels were negatively correlated with RFS of gastric cancer patients (Figure 1(b)). Therefore, the BGN expression level was negatively correlated with the prognosis of gastric cancer patients in a dose-dependent manner. In a stratified survival analysis according to the pathological stage, samples were restratified as BGN-high (equal or greater BGN levels than the median) and BGN-low (less BGN levels than the median), according to the expression levels of BGN mRNA. The HRs were 1.44 (95% CI 1.02-2.06, *p* = 0.038) and 2.16 (95% CI 1.22-3.87, *p* = 0.007) for high BGN expression in stages I-III (*n* = 365) and stage IV gastric cancer patients, respectively (Figures 1(c) and 1(d)). These results suggested that high BGN mRNA levels were significantly related to poor prognosis of gastric cancer patients.

### 3.2. Bioinformatics Analysis for the Gene and Protein Interaction Network of BGN

To understand the biological functions of BGN, we conducted bioinformatics analysis for genes coexpressed BGN on Oncomine. The analysis of genes coexpressed with BGN was conducted on Chen Gastric dataset [28]. We screened more than 10 genes with a strong correlation with BGN, such as THBS2, ARHGAP5, FN1, INHBA, and CDH11 (Figure 2(a)). Meanwhile, the bioinformatics analysis for the protein-protein interaction (PPI) network was conducted using STRING database (http://www.strig-db.org).  Figure 2(b) shows the PPI network of BGN; more than a dozen of genes were reported interacting with BGN through text mining, including genes like VCAN, TLR4, HSPG2, TGFB1, and GPC1. Most of the above genes were involved in cell growth, cell communication, signal transduction, and cell adhesion (Figure 2(c)), which was closely related to tumorigenesis.

### 3.3. GSEA of BGN in Gastric Cancer

To explore the cancer-related gene signatures of BGN, we performed a GSEA on the GSE26253 dataset, a downloaded microarray dataset of 432 gastric cancer cases. The expression of BGN was significantly associated with the following gene sets: Park hsc VS multipotent progenitors UP (Figure 3(a)), Nakamura metastasis model DN (Figure 3(b)), IVANOVA Hematopoiesis Stem Cell Long Term (Figure 3(c)), and RICKMAN Tumor Differentiated Moderately VS Poorly UP (Figure 3(d)) in GSE26253 dataset. GSEA results suggested that BGN was significantly enriched in gene signatures related to metastasis and poor prognosis, revealing that BGN might be associated with proliferation, poor differentiation, and high invasiveness of gastric cancer.

### 3.4. Prediction of Putative TFs of BGN by Bioinformatic Analysis

In order to further understand the carcinogenic mechanism, it is essential to explore the upstream regulation of BGN in gastric cancer. The TF prediction for BGN promoter region was processed using GTRD (http://gtrd.biouml.org/) and ALGGEN-PROMO databases (http://alggen.lsi.upc.es/cgi-bin/promo_v3/promo/promoinit.cgi?dirDB=TF_8.3). In Figure 4(a), the promoter region of BGN would be around the signal of H3K27Ac, which was located around the 1st exon and partially overlapped with CpG island. Meanwhile, the potential TFBSs were screened through GTRD and PROMO databases. By intersecting the two groups of gene sets, the eligible TFs were identified, including AR, CEBPA, CEBPB, E2F1, ELF1, GATA1, MAZ, PAX5, RXRA, SP1, STAT5A, TCF4, TP53, and YY1.  Figure 4(b) shows the location of these eligible TFBSs on the promoter of BGN. A linear regression analysis indicated that the expression of BGN was significantly and positively associated with TCF4 level, while negatively associated with AR or E2F1 (Figure 4(c)).

### 3.5. BGN Protein Level in Gastric Cancer Tissue

For gastric cancer, the protein expression level of BGN in tumor tissue was significantly higher than that in normal tissue (Figure 5). Unfortunately, BGN was mainly expressed in the extracellular matrix rather than in the intracellular matrix, which made quantitative analysis difficult.

## 4. Discussion

BGN, a member of the family of small leucine-rich repeat proteoglycans (SLRPs), is only considered as a component maintaining the structural integrity of extracellular matrix, involved in the regulation of inflammatory response, skeletal muscle development, and regeneration [9, 10]. In recent years, it has been gradually found that BGN is closely related to the occurrence and development of various malignant tumors, such as endometrial cancer [14], ovary cancer [15], pancreatic adenocarcinoma [16], esophageal squamous cell carcinoma [17], colorectal cancer [18], and prostate cancer [21]. In some malignant tumors, higher expression of BGN predicts more considerable invasiveness and worse prognosis [16, 17, 21, 22]. Therefore, it is valuable to reevaluate the prognostic significance and clinical meaning of BGN on other cancers.

A previous study has shown that BGN promotes tumor invasion and metastasis in gastric cancer both *in vitro* and *in vivo* and is associated with TNM stage. BGN plays an oncogenic role by activating the FAK signaling pathway in gastric cancer [19]. In this study, through analysis of public datasets (Figure 1(a)) and immunohistochemical analysis of tissue arrays (Figure 5), we confirmed that BGN expression was higher in tumor tissue than that in normal tissue. Unfortunately, since BGN was mainly distributed in the extracellular matrix, it cannot be quantified. Besides, we acquired a public microarray dataset, the GSE26253 dataset, containing 432 gastric cancer cases. Kaplan-Meier analysis of BGN for the RFS revealed that higher BGN expression level portended poorer prognosis in gastric cancer patients (*p* = 0.03). Stratification analysis showed that BGN was significantly associated with RFS of both stage I-III (*p* = 0.038) and stage IV (*p* = 0.007) patients with gastric cancer (Figure 1). Meanwhile, to explore the cancer-related gene signatures of BGN, we performed a GSEA on the GSE26253 dataset, revealing that BGN might be associated with poor proliferation, poor differentiation, and high invasiveness of gastric cancer. Also, we analyzed and predicted the potential TFs of BGN by bioinformatic analysis.

Limitations of this study included the following: (1) the protein expression levels of BGN could not be evaluated by immunohistochemistry (IHC) analysis. In gastric cancer tissue samples, the signal of BGN protein could only be seen in the extracellular matrix rather than in the intracellular matrix (Figure 5), which made it difficult for quantification. Meanwhile, (2) the mechanisms of BGN-associated aggressiveness and poor outcome of gastric cancer were still not clarified. (3) It needs to be further validated if BGN was a therapeutic target by experimental study.

Taken together, high BGN level could be enriched in gene signatures related to poor proliferation, poor differentiation, and high invasiveness. Kaplan-Meier analysis revealed that overexpression of BGN was significantly associated with poorer RFS in a dose-dependent manner in both stage I-III and stage IV gastric cancer patients. Therefore, BGN may be a potential prognostic and therapeutic biomarker for gastric cancer.

## Figures and Tables

**Figure 1:** BGN expression in gastric cancer tissue and prognostic value of BGN. (a) Differential expression of BGN between normal and gastric cancer tissue in the GSE65801 dataset. (b) Kaplan-Meier analysis of BGN and RFS in the GSE26253 dataset. The curves of red, green, blue, and brown represented Q1, Q2, Q3, and Q4 subgroups, respectively. Q1: 0 to 25% percentile; Q2: 25% to the median; Q3: the median to 75% percentile; Q4: 75% percentile to the maximum. (c) BGN impacts poor RFS on stage I-III and (d) stage IV gastric cancer patients from GSE26253 dataset.

**Figure 2:** Bioinformatics analysis for coexpressed genes and PPI network of BGN. The investigation was conducted on Oncomine and STRING websites. The interaction network of BNG was determined from curated database search, experiments, gene neighborhood, gene fusions, cooccurrence, text mining, coexpression, and protein homology. (a) Genes coexpressed with BGN in the Chen Gastric dataset. (b) PPI network of BGN. (c) The biological process of the related genes.

**Figure 3:** GSEA analysis of BGN. The expression of BGN was enriched in signatures of (a) Park hsc VS multipotent progenitors UP, (b) Nakamura metastasis model DN, (c) IVANOVA Hematopoiesis Stem Cell Long Term, and (d) RICKMAN Tumor Differentiated Moderately VS Poorly UP in GSE26253 dataset. As for heatmap of GSEA, columns are cases ranked by BGN expression, and rows are genes in the signature. Red represents the upregulated genes, and blue is the downregulated ones.

**Figure 4:** Prediction of putative TFs regulating BGN in gastric cancer. The prediction of BGN promoter region was processed using GTRD (http://gtrd.biouml.org/) and ALGGEN-PROMO (http://alggen.lsi.upc.es/cgi-bin/promo_v3/promo/promoinit.cgi?dirDB=TF_8.3) databases. The potential TFBSs were predicted by GTRD and ALGGEN-PROMO. (a) Overlapped TFs with sequence alignment and correlation significance were considered as eligible TFs. (b) The location of eligible TFBSs on the promoter of BGN. (c) Scatter plot of correlation between AR, E2F1, TCF4, and BGN expression levels.

**Figure 5:** Protein expression level of BGN in gastric cancer tissue was determined by immunohistochemical (IHC) staining. The representative images are (a) normal tissue and (b) cancerous tissue of gastric cancer.

**Table 1:** Summary of gene expression datasets of gastric cancer.

Accession no.	GSE26253	GSE65801
No. of patients	432	32
No. of healthy	0	32
Platforms^∗^	GPL8432	GPL14550
Country	South Korea	China
Date of study	2010-2019	2015-2016
Sex	N/A	Y
Clinical stage	Y	N/A
RFS months (range)	1.9-167.6	N/A

Platforms: GPL8432: Illumina HumanRef-8 WG-DASL v3.0. GPL14550: Agilent-028004 SurePrint G3 Human GE 8x60K Microarray (Probe Name Version).

## Data Availability

All the datasets used and analyzed during the current study are downloaded from NIH Gene Expression Omnibus (GEO) and ArrayExpress (https://www.ebi.ac.uk/arrayexpress/) which are available from the corresponding authors on reasonable request.

## Abbreviations

BGN: Biglycan
GSEA: Gene set enrichment analysis
RFS: Recurrence-free survival
HR: Proportional hazard ratios
CEA: Carcinoembryonic antigen
AFP: *α*-Fetoprotein
CA: Carbohydrate antigens
SLRPs: Small leucine-rich repeat proteoglycans
ECM: Extracellular matrix
95% CI: 95% confidence interval
TFBSs: Transcription factor binding sites
IHC: Immunohistochemistry
IRB: Institutional Review Board.

## References

[1] Kupfer S. S. (2017). Gaining ground in the genetics of gastric cancer. *Gastroenterology*.

[2] Siegel R. L., Miller K. D., Jemal A. (2018). Cancer statistics. *CA: A Cancer Journal for Clinicians*.

[3] Bray F., Ferlay J., Soerjomataram I., Siegel R. L., Torre L. A., Jemal A. (2018). Global cancer statistics 2018: GLOBOCAN estimates of incidence and mortality worldwide for 36 cancers in 185 countries. *CA: A Cancer Journal for Clinicians*.

[4] Power D. G., Kelsen D. P., Shah M. A. (2010). Advanced gastric cancer – slow but steady progress. *Cancer Treatment Reviews*.

[5] Hartgrink H. H., Jansen E. P. M., van Grieken N. C. T., van de Velde C. J. H. (2009). Gastric cancer. *The Lancet*.

[6] Sitarz R., Skierucha M., Mielko J. (2018). Gastric cancer: epidemiology, prevention, classification, and treatment. *Cancer Management & Research*.

[7] Tong W., Ye F., He L. (2016). Serum biomarker panels for diagnosis of gastric cancer. *Oncotargets & Therapy*.

[8] Schaefer L., Iozzo R. V. (2008). Biological functions of the small leucine-rich proteoglycans: from genetics to signal transduction. *Journal of Biological Chemistry*.

[9] Schaefer L., Babelova A., Kiss E. (2005). The matrix component biglycan is proinflammatory and signals through Toll-like receptors 4 and 2 in macrophages. *The Journal of clinical investigation*.

[10] Mercado M. L., Amenta A. R., Hagiwara H. (2006). Biglycan regulates the expression and sarcolemmal localization of dystrobrevin, syntrophin, and nNOS. *Faseb Journal Official Publication of the Federation of American Societies for Experimental Biology*.

[11] Nastase M. V., Young M. F., Schaefer L. (2012). Biglycan: a multivalent proteoglycan providing structure and signals. *Journal of Histochemistry & Cytochemistry Official Journal of the Histochemistry Society*.

[12] Berendsen A. D., Pinnow E. L., Maeda A. (2014). Biglycan modulates angiogenesis and bone formation during fracture healing. *Matrix Biology Journal of the International Society for Matrix Biology*.

[13] Myren M., Kirby D. J., Noonan M. L. (2016). Biglycan potentially regulates angiogenesis during fracture repair by altering expression and function of endostatin. *Matrix Biology*.

[14] Liu Y., Li W., Li X. (2014). Expression and significance of biglycan in endometrial cancer. *Archives of Gynecology & Obstetrics*.

[15] Pan S., Cheng L., White J. T. (2009). Quantitative proteomics analysis integrated with microarray data reveals that extracellular matrix proteins, catenins, and P53 binding protein 1 are important for chemotherapy response in ovarian cancers. *Omics A Journal of Integrative Biology*.

[16] Aprile G., Avellini C., Reni M. (2013). Biglycan expression and clinical outcome in patients with pancreatic adenocarcinoma. *Tumor Biology*.

[17] Zhu Y. H., Yang F., Zhang S. S., Zeng T. T., Xie X., Guan X. Y. (2013). High expression of biglycan is associated with poor prognosis in patients with esophageal squamous cell carcinoma. *International Journal of Clinical & Experimental Pathology*.

[18] Gu X., Ma Y., Xiao J. (2012). Up-regulated biglycan expression correlates with the malignancy in human colorectal cancers. *Clinical & Experimental Medicine*.

[19] Hu L., Duan Y. T., Li J. F. (2014). Biglycan enhances gastric cancer invasion by activating FAK signaling pathway. *Oncotarget*.

[20] Sun H., Wang X., Zhang Y. (2016). Biglycan enhances the ability of migration and invasion in endometrial cancer. *Archives of Gynecology and Obstetrics*.

[21] Jacobsen F., Kraft J., Schroeder C. (2017). Up-regulation of biglycan is associated with poor prognosis and PTEN deletion in patients with prostate cancer. *Neoplasia*.

[22] Schulz G. B., Grimm T., Sers C. (2019). Prognostic value and association with epithelial-mesenchymal transition and molecular subtypes of the proteoglycan biglycan in advanced bladder cancer. *Urologic Oncology*.

[23] Lee J., Sohn I., do I. G. (2014). Nanostring-based multigene assay to predict recurrence for gastric cancer patients after surgery. *PLoS One*.

[24] Li H., Yu B., Li J. (2015). Characterization of differentially expressed genes involved in pathways associated with gastric cancer. *PLoS One*.

[25] Subramanian A., Tamayo P., Mootha V. K. (2005). Gene set enrichment analysis: a knowledge-based approach for interpreting genome-wide expression profiles. *Proceedings of the National Academy of Sciences of the United States of America*.

[26] Ding J., Kuo M. L., Su L. (2017). Human mitochondrial pyrroline-5-carboxylate reductase 1 promotes invasiveness and impacts survival in breast cancers. *Carcinogenesis*.

[27] Halstensen T. S., Scott H., Brandtzaeg P. (1990). Human CD8+ intraepithelial T lymphocytes are mainly CD45RA−RB+ and show increased co-expression of CD45R0 in celiac disease. *European Journal of Immunology*.

[28] Chen X., Leung S. Y., Yuen S. T. (2003). Variation in gene expression patterns in human gastric cancers. *Molecular Biology of the Cell*.

[29] Hu S., Li P., Wang C., Liu X. (2020). *Prognostic Value of Biglycan in Gastric Cancer*.

